# An Improved Brain MRI Classification Methodology Based on Statistical Features and Machine Learning Algorithms

**DOI:** 10.1155/2021/8608305

**Published:** 2021-12-07

**Authors:** Muhammad Fayaz, Muhammad Shuaib Qureshi, Karlygash Kussainova, Bermet Burkanova, Ayman Aljarbouh, Muhammad Bilal Qureshi

**Affiliations:** ^1^Department of Computer Science, University of Central Asia, Naryn 722918, Kyrgyzstan; ^2^Department of Computer Science and IT, University of Lakki Marwat, Lakki Marwat 28420, KPK, Pakistan

## Abstract

In this paper, we have proposed a novel methodology based on statistical features and different machine learning algorithms. The proposed model can be divided into three main stages, namely, preprocessing, feature extraction, and classification. In the preprocessing stage, the median filter has been used in order to remove salt-and-pepper noise because MRI images are normally affected by this type of noise, the grayscale images are also converted to RGB images in this stage. In the preprocessing stage, the histogram equalization has also been used to enhance the quality of each RGB channel. In the feature extraction stage, the three channels, namely, red, green, and blue, are extracted from the RGB images and statistical measures, namely, mean, variance, skewness, kurtosis, entropy, energy, contrast, homogeneity, and correlation, are calculated for each channel; hence, a total of 27 features, 9 for each channel, are extracted from an RGB image. After the feature extraction stage, different machine learning algorithms, such as artificial neural network, *k*-nearest neighbors' algorithm, decision tree, and Naïve Bayes classifiers, have been applied in the classification stage on the features extracted in the feature extraction stage. We recorded the results with all these algorithms and found that the decision tree results are better as compared to the other classification algorithms which are applied on these features. Hence, we have considered decision tree for further processing. We have also compared the results of the proposed method with some well-known algorithms in terms of simplicity and accuracy; it was noted that the proposed method outshines the existing methods.

## 1. Introduction

The human brain is one of the unsolved mysteries of science. Its complexity has perplexed and vexed scientists till today. It contains over 85 ± 8 billion neurons with an equal number of nonneuronal cells. Brian controls and coordinates our body movements, homeostasis–body temperature, heart rate, blood pressure, and fluid balance. It is responsible for our emotions, fight or flight mood, memory, cognition, motor learning, and learning, remembering, and communicating processes [1]. The brain is a network of nerve cells that grow, build new synapsis, and die continuously, but the abnormal and uncontrolled growth of nerve cells leads to the formation of tumors. Brain tumors can be also caused by abnormal activity of other body parts like the lungs, breast, and skin [2]. Brain tumor is one of the most fatal causes of cancer-related deaths in the world. According to the most recent report by the Central Brain Tumor Registry of the United States, there were 81,246 deaths attributed to primary malignant brain and other central nervous system (CNS) tumors for the period of 2013-2017. On average, there are 16,249 deaths per year, and the survival rate after diagnosis of a primary malignant brain and other CNS was 36%, lowest in 40+ age groups (90.2%), while in age group 0-14 years, survival rates were 97.3% [3].

Classification of normal and abnormal brain images obtained from MRI is the first step towards tackling the staggering deaths caused by brain tumors. However, the large amount of data from MRI makes their manual classification tedious, error-prone, and time-consuming and requires an expert. The observer faces a great difficulty in analyzing and interpreting the images and detecting the tumor [4]. Hence, it is necessary to develop and implement an automatic image analyzing system. It should be faster and accurate in its inferences of the MRI images, and it should be easy to use. Research has been done in this area and in literature; we have a wide variety of automatic and accurate medical diagnostic techniques introduced by applying complex signal/image processing methods which use the computational intelligent techniques of machine learning algorithms. MRI image processing methods are categorized into two types. One is supervised classification, which exploits the algorithms like artificial neural network (ANN), *k*-nearest neighbor (kNN), and support vector machine (SVM). The other is unsupervised classification where methods of Self-Organization Map (SOM) and fuzzy *c*-means are employed. The supervised classification gives more accurate results as compared to unsupervised classification methods [5]. These techniques help doctors with diagnosis during presurgical and postsurgical procedures [4].

The information from MRI images can be analyzed and processed using supervised or unsupervised algorithms and can be categorized into normal or abnormal classes. But the accuracy of the categorization depends on how we extract the features from the images and how relevant the features are to determine the disorder. Some widely used methods include the Fourier transform-based techniques, independent component analysis (ICA), wavelet transform-based techniques [6, 7], and statistical feature extraction methods like kurtosis, skewness, quartiles, mode, median, mean, and standard deviation [8]. It is important to extract the meaningful features, but it also increases the computational burden of the classifier, so to balance the drawbacks, the best option is to choose a feature extraction method, which can determine the fewer most relevant features as possible to get the complete characteristic anatomy of the tumor hence, reducing the extra computational complications for unnecessary feature extraction. Keeping the constraints under view, one of the suitable methods is wavelet transform, which is a nonstatistical method. It provides the local frequency information and detailed coefficients of the image at various levels. Employing principal component analysis (PCA) with wavelet transform reduces the dimensions and overcomes the computational complexity [9]. Moreover, wavelet transform is good for getting frequency space information from nonstationary images; it is also amenable to computer-based analysis—the analysis can be monitored and controlled by changing the wavelets in the selected sequence [5]. In our work, we applied the methodology as image processing, feature extraction, feature reduction, and finally classification of the brain tumor.

As more useful, the feature extraction is, similarly, the challenging task it gets. Several studies have used different methods for feature extraction. For instance, Gabor feature, discrete wavelet transform, spectral mixture analysis, texture feature, principal component analysis, minimum noise fraction transform. By dimensionality reduction, we can have our focus on only few key features. The widely implemented algorithms for feature reduction are independent component analysis, principal component analysis, linear discriminant analysis, and genetic algorithms [4].

After features extraction stage, classification of the images is done. In classification stage—classification of the images into normal/abnormal or tumor/not tumor classes. The classifier takes the purified images with selected features for training and testing. Various classifiers—each having pros and cons—have been used as discussed above like *k*-nearest neighbor (kNN), support vector machine (SVM), artificial neural network (ANN), Hidden Markov Model (HMM), and the Probabilistic Neural Network (PNN). The common application of these algorithms can be found in handwritten digit identification, text classification, face identification, object detection and recognition, and speaker identification for medical purposes [4]. Classification has two parts—training and testing. Firstly, for training, the already labeled and known data is given to the algorithm. The algorithm gets trained on these data and builds the model to predict/classify the unknown data. Secondly, the test data which is the unknown data is given to the classifier algorithm after training has been done. After this part, the performance of the algorithm is evaluated. The error in classification or the precision of the classifier depends on the efficient training. Usually, more training data helps the classifier to get tuned and build a more feasible or general model. As analyzing human MR images of the brain manually is slow, expensive, labor-intense, and error-prone, we are proposing the accurate, automatic analyzing, and robust classification of human MR images of the brain.

Many researchers have proposed different types of approaches for brain MRI classification. A study by Chaplot et al. [6] compared the self-organizing maps and support vector machine for the classification of MR images of brain tumor into normal and abnormal. Using wavelets as inputs to neural network SOM and SVM, they concluded that SVM has a better classification rate (98%) than SOM (94%). Feature extraction was done using a two-dimensional discrete wavelet transform and Daubechies filters were used for the decomposition. Maitra and Chatterjee [10] used a unique and improved version of an orthogonal discrete wavelet transform for feature extraction—the Slantlet transform; this transform gave an improved time localized space information for nonstationary MRI images. Applying an improved feature extraction method provided a better feature vector to be used for the training of the backpropagation neural network-based binary classifier they employed—it classified normal brain images and images of patients with Alzheimer with 100% accuracy. El-Dahshan et al. [11] introduced a hybrid technique with three stages—feature extraction, dimensionality reduction, and classification—to classify MRI brain tumor images. Discrete wavelet transformation (DWT) was used in the feature extraction stage; principal component analysis (PCA) was used in dimensionality reduction stage to focus on more essential features of MRI images. Then, two classifiers, namely, feed-forward back-propagation artificial neural network (FA-ANN) and kNN, have applied for the classification of the subject MRI images into normal and abnormal images. The results for FA-ANN were 97% accurate while for kNN, the accuracy was calculated to 98%. Furthermore, Zhang et al. [12] also proposed a three-stage classification of brain images. Zhang et al. followed the same methods as El-Dahshan, but they used the Scaled Conjugate Gradient (SCG) in Back-propagation Neural Networks to get the optimal weights. The accuracies for training and testing images were 100% (66 images), while the computational time for each image was only 0.0451 s. A similar approach was adopted by Fayaz et al. [13] with the preprocessing stage, feature extraction stage, and finally classification stage. Using median filter, the noise from MRI grayscale images was removed in the preprocessing stage and converted into RGB colored images. During feature extraction stage, the red, green, and blue channels were extracted from RGB images; for each channel, the mean, variance, and skewness are also calculated. Then, using kNN, the final classification was carried out. An accuracy of 98% training and 95% test data was obtained for normal images while 100% training and 90% test accuracy for abnormal images was obtained.

Different methodologies have been proposed by different authors for classification in different areas, such as Alotaibi et al. [14] who proposed a hybrid method based on convolutional neural network (CNN) and long short-term memory (LSTM) recurrent neural network for classification of text into psychopath or nonpsychopath classes. The results indicate that this method provides good results. Similarly, another method has been proposed by Hussain et al. [15] for depression classification in social media by using deep learning method.

In this paper, a novel method based on machine learning algorithms and statistical features has been proposed. The main aim of this paper is twofold, first to reduce the computation time and second to increase the accuracy for brain MRI classification. The main contributions of this paper are below:

- The grayscale images are converted to RGB images, and red, green, and blue channels are then extracted from RGB images. The histogram equalization has been applied on each channel of RGB images in order to enhance the quality of these channels
- A novel method has been proposed to extract statistical features, namely, mean, variance, skewness, kurtosis, entropy, energy, contrast, homogeneity, and correlation from red, green, and blue channels of RGB images and concatenated to feed to the machine learning algorithms to classify the brain MRI images into normal and abnormal
- In the proposed method, we have applied different classification algorithms, such as *k*-nearest neighbor, decision tree, random forest, and Naïve Bayes to select an algorithm with the highest accuracy on the extracted features

The structure of the remaining paper is organized as follows: in Section 2, the proposed methodology is explained in detail; Section 3 is about implementation, results, and discussion. The conclusion is given in the last stage.

## 2. Proposed Methodology

In this work, we have proposed a novel method for brain MRI classification. The proposed model consists of four stages, namely, preprocessing, feature extraction, classification, and performance evaluation. The conceptual model of the proposed model is depicted in Figure 1.

The detailed schematic diagram of the proposed methodology is shown in Figure 2. In the preprocessing stage of the proposed model, the median filter has been used to remove salt-and-pepper noise from MRI images. Usually, the MRI images are affected by salt-and-pepper noise and median filter is the most common filter used for removing such type of noise from MRI images [13, 16].

In the preprocessing stage, the original grayscale brain images have been converted to RGB images, and red, green, and blue channels are extracted from the RGB images. The next operation that is deployed on the images in the preprocessing module is histogram equalization. The histogram equalization is applied on each channel of the RGB images to improve the quality of these images and make them able to be used for further processing. In next feature extraction module of the proposed model, the statistical features have been calculated for red, green, and blue channels with the purpose to handle the curse of dimensionality.

These features are stored and combined in a file and labeled to train the machine learning algorithms. In the classification module, we have applied different machine learning algorithms, such as artificial neural network, *k*-nearest neighbor algorithm, naïve Bayes classifier, random forest, and decision tree classifier for classification, and the extracted features are given as inputs to these classifiers. In the classification module, we have used the percentage split method to divide the data into training and testing. In the performance evaluation module first, we have the classification algorithms by using different metrics, such as precession, recall, and *F*_1_-score.

### 2.1. Preprocessing

There are three stages that make up the proposed methodology: preprocessing, feature extraction, and classification and performance evaluation as illustrated in Figure 2. Each stage consists of several steps, where preprocessing includes noise removal, grayscale to RGB conversion, and histogram equalization.

In the preprocessing stage, the images from a dataset of 140 samples are first issued for noise removal. Different types of noises exist in different image modalities, such as spackle noise, Gaussian noise, and salt-and-pepper noise. To remove these noises from images, different types of filters are used, such as Wiener filter, mean filter, and median filter. The MRI images are normally affected by salt-and-pepper noise, and the most effective and commonly used filter for this type of noise is median filter [16, 17].

A median filter can sharpen the images without disturbing the edges. In the proposed work, we have used the median with a window size 3 × 3 to remove salt-and-pepper noise from the images and smooth the images. Consequently, the grayscale images are converted to RGB for further processing, as illustrated in Figure 3. The necessity of conversion of the grayscale image into a color image is in its detailed representation of pixels. After converting the grayscale image into RGB, it is possible to represent it in red, blue, and green channels. This allows us to extract features from different points of view and then see a more detailed analysis of the anomalies in the brain.  Figure 4 illustrates the way a simple RGB image is converted into three channels (red, green, and blue).

In the proposed work, we have also used histogram equalization, which is the last step in the preprocessing stage, where it is used as a technique to adjust the image intensity for contrast enhancement [18]. In this work, we have used the histogram equalization to enhance the quality of red, green, and blue channels of an RGG image. The theoretical background of the histogram equalization is given in detail here. Assume there is a matrix of integer pixels that has a range from 0 to L − 1, and *f* is an image that is represented as a m(r) by m(c) matrix. In this case, *L* is the value/number of all possible values of the intensities (usually, *L* is equal to 256). And *p* is denoted as a normalized histogram of *f* as defined in equation (1), with a particular bin for each intensity. So, *g*, which is an equalized histogram image, is defined as in equation (2).

(1) $$\begin{array}{c} \;P\left(n\right)=\frac{\text{Number of pixels with intensity }n}{\text{ Total number of pixels }}, \end{array}$$

(2) $$\begin{array}{c} g\left(i,j\right)=\text{floor}\left(\;\left(L-1\right)\;\overset{f\left(i,j\right)}{\underset{n=0}{\sum }}p\left(n\right)\right). \end{array}$$

Here, floor () function is used to round down to the nearest integer value. This is the same as transforming pixel intensities *k*, by the *f* function defined in equation (3). A given transformation appears from an idea of the intensities of the *f* and *g* functions as continuous random variables *X* and *Y* on the range from 0 to *L* − 1, where *Y* is defined as in equation (4).

(3) $$\begin{array}{c} Y=T\left(X\right)=\left(L-1\right)\int_{0}^{x}p\left(x\right)dx, \end{array}$$

(4) $$\begin{array}{c} g\left(i,j\right)=\text{floor}\left(\;\left(L-1\right)\;\overset{f\left(i,j\right)}{\underset{n=0}{\sum }}p\left(n\right)\right), \end{array}$$

where *p*(*x*) is the probability density function (PDF) and *T* is the cumulative distributive function. We also assume here that *T* is differentiable and is an invertible function. Consequently, *Y*, which is defined by *T*(*X*) in this context, is distributed uniformly, namely, that *p*(*y*) = 1/(*L* − 1). These are defined in equation (5) and equation (6).

(5) $$\begin{array}{c} \frac{d}{dY}T\;\left(T^{-1}\left(y\right)\right)=\frac{d}{dy}y=1, \end{array}$$

(6) $$\begin{array}{c} py\left(y\right)=\frac{1}{L-1}. \end{array}$$

### 2.2. Feature Extraction

An original image (512 × 512 = 134,217,728) has an excessive number of pixels, and if these numbers of features are directly fed to machine learning algorithms, then it is impossible to compute in polynomial time. In the feature extraction stage, the features obtained in the proposed work, we have extracted some informative features from each channel of the RGB image. The first four statistical moments, namely, mean, variance, skewness, and kurtosis, and cooccurrence matrix features, namely, entropy, energy, inverse difference, and correlation, have been calculated of the approximate images obtained in the feature extraction stage [19]. In equations (7)–(10), mean, variance, skewness, and kurtosis have been represented, respectively. Mean is used to describe the bright mean and dark mean in an image. Variance is used to describe the contrast of the image. Skewness is a measure of symmetry, and kurtosis is used to measure the peak and flatness relative to a normal distribution.

(7) $$\begin{array}{c} \text{Mean }=\frac{\sum_{i=1}^{N}p_{i}}{N}, \end{array}$$

(8) $$\begin{array}{c} \text{Variance}=\frac{\;\sum_{i=1}^{N}{\left(p_{i}-\bar{p}\right)}^{2}}{n}, \end{array}$$

(9) $$\begin{array}{c} \text{Skewness}=\frac{\sum_{i=1}^{N}{\left(p_{i}-\bar{p}\right)}^{3}}{n}, \end{array}$$

(10) $$\begin{array}{c} \text{Kurtosis}=\frac{\sum_{i=1}^{N}{\left(p_{i}-\bar{p}\right)}^{4}}{N}, \end{array}$$

where *N* represents the number of pixels in total in an image; the mean of an image pixel values is represented by $\bar{p}$. The calculation of energy, correlation, entropy, contrast, and homogeneity has been done in equations (11)–(15), respectively.

(11) $$\begin{array}{c} \text{Eng}=\underset{i}{\sum }\underset{j}{\sum }{\left(\Omega_{i,j}\right)}^{2}, \end{array}$$

(12) $$\begin{array}{c} \text{Corr}=\frac{1}{\sigma_{\alpha }\sigma_{\beta }}\underset{m}{\sum }\underset{n}{\sum }\left(p-{\bar{p}}_{\alpha }\right)\left(\left(p-{\bar{p}}_{\beta }\right)\right.\Omega_{i,j}, \end{array}$$

(13) $$\begin{array}{c} \text{Ent}=-\underset{m}{\sum }\underset{n}{\sum }\Omega_{i,j}\log_{2}\Omega_{i,j}, \end{array}$$

(14) $$\begin{array}{c} \text{Cont}=\underset{i}{\sum }\underset{j}{\sum }{\left(\Omega_{i,j}\right)}^{2}{\left(i-j\right)}^{2}, \end{array}$$

(15) $$\begin{array}{c} \text{Homog}=\underset{i}{\sum }\underset{j}{\sum }\frac{\Omega_{i,j}}{\left|i-j\right|}, \end{array}$$

where Eng, Corr, Ent, Cont, and Homog represent energy correlation, entropy, contrast, and homogeneity, respectively.

In the proposed work, we have calculated nine features, namely, mean, variance, skewness, kurtosis, entropy, correlation, entropy, energy, contrast, and energy for red, green, and blue channels, respectively, in the feature extraction stage. The graphical representation of the feature extraction stage is illustrated in Figure 5. We have then combined these features in a file and have been fed to a classifier to classify the brain MRI images into normal or abnormal.

In the classification stage, two cases have been considered: the percentage split method has been used in which the whole data is divided into two datasets, namely, training and testing as visualized in Figure 6.

### 2.3. Classification

Artificial neural network performance is better as compared to counterpart algorithms for complex data [4, 19, 20]. The explanation of MLP is given below. The sum of products of weights and neuron values and bias is done using the below equation:

(16) $$\begin{array}{c} \emptyset_{m}=\overset{r}{\underset{n=1}{\sum }}P_{mn}l_{m}+\beta_{m}, \end{array}$$

where *r* indicates number of inputs, input variables is presented by *l*_*m*_, *β*_*m*_ represents the bias, and *P*_*mn*_ indicates weights. A set of activation functions are available that we can apply to hidden layer neurons.

Sigmoid, tangent hyperbolic sigmoid, and ReLU activation functions are donated in equations (17), (18), and (19) correspondingly.

(17) $$\begin{array}{c} \text{Sigmoid}=\frac{1}{1+e^{\emptyset_{m}}}, \end{array}$$

(18) $$\begin{array}{c} \tan h=\frac{e^{{-\emptyset }_{m}}-e^{{-\emptyset }_{m}}}{e^{-\emptyset_{m}}+e^{-\emptyset_{m}}}, \end{array}$$

(19) $$\begin{array}{c} \text{ReLU}=\max\left(0,\emptyset_{m}\right). \end{array}$$

The mean, variance, skewness, kurtosis, entropy, correlation, energy, contrast, and homogeneity features calculated in the feature extraction stage for each channel of the RGB image and combined are fed to the artificial neural network. By applying an activation *ψ*_*q*_ function on ∅_*m*_, the output of a partial neuron can be obtained as in the following equation:

(20) $$\begin{array}{c} \psi_{q}=\psi_{q}\;\left[\overset{k}{\underset{p=1}{\sum }}p_{mn}l_{m}+\beta_{m}\right]. \end{array}$$

The structure diagram of the proposed artificial neural network used in the proposed model is given in Figure 7.

The second algorithm that we have used in the proposed work for brain MRI classification based on the features extracted in feature extraction stage is decision tree classifier. Decision tree classifier is known as one of the most widespread methods in mining data used for classification purposes. It is based on varieties of classes for developing prediction models. This algorithm is used to classify a dataset into subtrees that make up a global inverted tree (consisting of the root, internal, and leaf nodes). An algorithm is efficient for huge and complicated datasets. In case the dataset is sizable, training data is divided into validation states [21]. Decision trees are basically illustrated graphically as a hierarchically represented graph. This diagram includes branches and a starting node (root node) [22]. Branches (conditions) are known to be a group of nodes interconnected and inherited some properties from one another that should lead to a final decision (classification class) [22]. To build branches that are based on conditions, a variety of splitting criteria are used. The most used are Gain Ratio and Gini Index [23]. When it comes to Gain Ratio, decreasing the irregularity of every node leads to the tree height reduction which is an aim of the algorithm. Irregularity is defined as in the following equation:

(21) $$\begin{array}{c} I=-\underset{c}{\sum }p\left(c\right)\;\log_{2}p\left(c\right). \end{array}$$

Here, *p*(*c*) is a portion of the data belonging to the *c* class. This way, the feature with the maximum Gain Ratio is defined as a tree root (see the following equation).

(22) $$\begin{array}{c} \text{Gain}\left(A\right)=I-I\left(\text{res}\right). \end{array}$$

Here, *I*(res) is known as irregularity at all of the classes at the moment when a particular feature was used. It is computed as in the following equation:

(23) $$\begin{array}{c} I\left(\text{res}\right)=-\underset{v}{\sum }p\left(v\right)\underset{c}{\sum }p\left(\text{c}\;|\;v\right)\log_{2}p\left(c\;|\;v\right). \end{array}$$

Gini Index is basically defined as the split measure and computed as in the following equation:

(24) $$\begin{array}{c} I\left(\text{Gini}\right)=1-\underset{j}{\sum }p{\left(cj\right)}^{2} \end{array}$$

Here, *p*(*c*) represents the relative frequency of cases that belong to the *cj* class. Then, the information gain is computed as in the following equation:

(25) $$\begin{array}{c} G=I-\sum \frac{cj}{c}\;I\left(c\right). \end{array}$$

A splitting feature is then chosen to maximize the Gini Index.

The third algorithm that we have used in the proposed work for brain MRI classification based on the features extracted in feature extraction is random forest (RF). Random forest classification implies decision tree (DT) algorithm as its base. In the case of random forest, we assume that the system is already familiar with the single tree classifier and consists of a large number of them. Therefore, to examine where the input value belongs, it should go through each of the single trees made from the DTAs. After the processing is finished, each of the trees gives an output, which scientists call “votes,” and the class that had the most votes is shown as a result. The mandatory rules to follow while constructing each of the trees [24] are as follows:

- If the number of the features of the training set is *N*, each tree must have a smaller number of features that are chosen randomly from the set. The subsets which construct the tree are gathered with replacement from the main features
- During tree growth, it is important not to overburden the depth of the tree to conclude accurate results
- The largest extent should be achieved in each tree; there is no place for pruning

In RF, the correlation between the trees defines the error rate, which means that the increase of the correlation between the feature trees grows the error rate as well. Therefore, to avoid it, an individual tree should be a strong classifier and should have its feature strength. This algorithm does not require any cross-validation or any separated tests to estimate if the result is biased or unbiased [25].

The fourth algorithm that we have used in the proposed work for brain MRI classification based on the features extracted in feature extraction is Naïve Bayes classifier. Based on strong assumptions of the independence of varieties in Bayes theorem, Naïve Bayes is an algorithm for classification purposes. The algorithm assumes that the variables are independent of each other, Gaussian distribution of numeric predictors with mean and standard deviation computed from the training dataset. The given algorithm is normally used as an alternative for decision trees, though compared to those, it skips any instance of the dataset with null (N/A) values [26].

In probabilities, Naïve Bayes is known to be a probabilistic classifier. In other words, in the dataset *d*, all classes *c* ∈ *C*, the class of *c* that has the maximum posterior probability in the abovementioned dataset (*ĉ* is the estimate of the correct class) (see the following equation).

(26) $$\begin{array}{c} \hat{\text{c}}=\text{argmax }P\left(c\;|\;d\right). \end{array}$$

The major idea of the Bayesian classification is to change equation (26) to other probabilities.

(27) $$\begin{array}{c} P\left(x\;|\;y\right)=\frac{P\left(y\;|\;x\right)\;P\left(x\right)}{P\left(y\right)} \end{array}$$

might be transformed to the following equation:

(28) $$\begin{array}{c} \hat{\text{c}}=\text{argmax }P\left(c\;|\;d\right)=\text{argmax}\left(\frac{P\left(d\;|\;c\right)P\left(c\right)}{P\left(d\right)}\right). \end{array}$$

If we drop the denominator *P*(*d*), equation (28) might be easily simplified. Since *P*(*d* | *c*)*P*(*c*)/*P*(*d*) is computed for every possible class, the formula can be simplified conveniently. However, *P*(*d*) is not changed for every class; we concentrate on the class that is most probable for the same *d* that must present an identical *P*(*d*) of probability [39, 40]. Therefore, the class that maximizes equation (29) can be chosen:

(29) $$\begin{array}{c} \hat{\text{c}}=\text{argmax }P\left(c\;|\;d\right)p\left(d\right)=\text{argmax }P\left(d\;|\;c\right)\;P\left(c\right). \end{array}$$

The fourth algorithm that we have used in the proposed work for brain MRI classification based on the features extracted in feature extraction is KNN classifier.

*k*-nearest neighbor (KNN) is a widely spread machine learning algorithm that is used for classification purposes. It is commonly used for pattern recognition where data samples are classified based on the nearest neighbor of the class; they might belong to [27, 28]. *k*-nearest neighbor (KNN) is a simple algorithm, which stores all cases and classify new cases based on similarity measure KNN algorithm also called as (1) case-based reasoning, (2) *k*-nearest neighbor, (3) example-based reasoning, (4) instance-based learning, (5) memory-based reasoning, and (6) lazy learning [29].

For performance measurements, we have used different performance evaluators such as precession, recall, and *F*_1_-score [13, 19] to measure the performance of the proposed approach.

## 3. Implementation, Results, and Comparative Analysis

### 3.1. Implementation Setup

In this section, we have briefly discussed the implementation details. The entire implementation of the proposed work is done in Python installed on Intel(R) Core (TM) i7-7500U having NVIDIA GeForce 940MX GPU, 15 GB DDR2 RAM. In the proposed work, some libraries of Python like NumPy, Keras, SciPy, and Sklearn are used for model building and classification purposes.

In this study, we have considered T2-weighted MRI of 512 × 512 size images taken from the Harvard University medical website [30]. A sample image from each disease is shown in Figure 8, along with a normal brain MRI.

In the proposed work, we have applied different algorithms, such as artificial neural network, decision tree, naïve Bayes, and KNN and have applied on the data collected in the feature extraction stage. The performance evaluation results for each algorithm are given in detail in terms of confusion matrix, precision, recall, and *F*_1_-score.

### 3.2. Results

A structure diagram of the implemented neural network is exhibited in Figure 9 and the corresponding specifications are listed in Table 1. The confusion matrix for classification results obtained through ANN is illustrated in Figure 10. The confusion shows that out of 42 abnormal images, the ANN accuracy classified 29 images and inaccurately classified 2 images. Similarly, out of 42 normal images, the ANN classified 8 images correctly. The precision, recall, and *F*_1_-score are calculated for ANN classification results and are listed in Table 2. Also, you can see the visualization of the performance evaluation in Figure 11.

The confusion matrix for classification results obtained through random forest is illustrated in Figure 12. The confusion shows that out of 42 abnormal images, the random forest accuracy classified 24 images and inaccurately classified 2 images. Similarly, out of 42 normal images, the random forest classified 9 images correctly. The precision, recall, and *F*_1_-score are calculated for random forest classification results and are listed in Table 3. Also, you can see the visualization of the performance evaluation in Figure 13.

The confusion matrix for classification results obtained through Naïve Bayes is illustrated in Figure 14. The confusion shows that out of 42 abnormal images, the Naïve Bayes accuracy classified 20 images and inaccurately classified 2 images. Similarly, out of 42 normal images, the Naïve Bayes classified 9 images correctly. The precision, recall, and *F*_1_-score are calculated for Naïve Bayes classification results and are listed in Table 4. Also, you can see the visualization of the performance evaluation in Figure 15.

The confusion matrix for classification results obtained through the *k*-nearest neighbor algorithm is illustrated in Figure 16. The confusion shows that out of 31 abnormal images, the KNN accuracy classified 24 images and inaccurately classified 7 images. Similarly, out of 11 normal images, the KNN classified 11 images correctly. The precision, recall, and *F*_1_-score are calculated for KNN classification results and are listed in Table 5. Also, you can see the visualization of the performance evaluation in Figure 17.

The confusion matrix for classification results obtained through decision tree classifier is illustrated in Figure 18. The confusion matrix shows that out of 42 abnormal images, the decision tree classifier accurately classified 39 images and inaccurately classified 0 images. Similarly, out of 42 normal images, the decision tree classifier classified 17 images correctly. The precision, recall, and *F*_1_-score are calculated for decision tree classifier classification results and are listed in Table 6. Also, you can see the visualization of the performance evaluation in Figure 19.

### 3.3. Comparative Analysis

We have applied different machine learning algorithms in the classification stage on the features obtained in the feature extraction stage. The results indicate that classification and regression tree performance is better when we apply it to the extracted features; hence, we have considered this classification and recorded the results and compared with some well-known classification methods as listed in Table 7. We have compared the proposed method with some other methods in order to measure the performance of the proposed method. The selection norms of the qualified algorithms are simplicity, computation complexity, and accuracy. The results exhibit that the proposed method has outshined the other algorithms.

## 4. Conclusion

Accurate classification of brain MRI images with a small dataset is challenging. Normally, two types of strategies are used to classify the brain MRI images, firstly to apply deep learning algorithms, such as convolutional neural network to classify the brain MRI image, but the problem with deep learning is that it requires an immense number of images to train the model. In the case of convolutional neural network, the whole image is given as input to the algorithm. Secondly, if we have a small set of images then usage of convolution of neural network is not a wise choice because convolutional neural network performs worst on a small dataset. Hence, the next choice is to apply a simple machine learning algorithm, such as an artificial neural network with one or two hidden layers, *k*-nearest neighbor algorithm, decision tree, etc., but the problem with these algorithms is that we cannot feed complete image to these algorithms because it requires a lot of computation time. Hence, proper feature engineering is required to reduce the curse of dimensionality and to extract some features of interest from images. For this purpose, in the proposed work, a novel method has been applied for extracting features of interest from images. First, the grayscale images are converted to RGB images and red, green, and blue channels are then extracted from RGB images. The histogram equalization has been applied on each channel of RGB images in order enhance the quality of these channels. Then, statistical parameters have been calculated for red, green, and blue channels of RGB images. A total of 27 (9 + 9 + 9) features are extracted for each image, and features for all images are then stored in a file and labeled accordingly to train the machine learning algorithms. We have applied different machine learning algorithms, random forest, ANN, KNN, naïve Bayes, and decision tree, on the features extracted in the feature extraction stage. The performance measures indicate that the performance of the decision tree is far better as compared to the counterpart algorithms. The proposed model is also compared with some state-of-the-art algorithms, and the results exhibit that the performance of the proposed method is far better as compared to other counterpart algorithms.

The limitation of the proposed method is that we have applied this method only on a small dataset that has 140 images and have not applied it on a large dataset.

## Figures and Tables

**Figure 1:** Abstract diagram of the proposed model.

**Figure 2:** Detailed schematic diagram of the proposed methodology for brain MRI classification.

**Figure 3:** (a) Grayscale image and (b) RGB image.

**Figure 4:** An RGB image and its three channels (red, green, and blue).

**Figure 5:** Visualization of feature extraction mechanism in the feature extraction stage.

**Figure 6:** Visualization of the division of data into training and testing by using the percentage split method.

**Figure 7:** Structure diagram of the ANN used in the proposed work.

**Figure 8:** (a) Normal brain MRI, (b) glioma, (c) meningioma, (d) Alzheimer, (e) Alzheimer plus, (f) visual agnosia and pick's disease, (g) sarcoma, and (h) Huntington's disease.

**Figure 9:** Implemented neural network.

**Figure 10:** Confusion matrix for ANN classifier.

**Figure 11:** Graphical representation of Table 2.

**Figure 12:** Confusion matrix for random forest classifier.

**Figure 13:** Graphical representation of Table 3.

**Figure 14:** Confusion matrix for Naïve Bayes classifier.

**Figure 15:** Graphical representation of Table 4.

**Figure 16:** Confusion matrix for KNN classifier.

**Figure 17:** Graphical representation of Table 5.

**Figure 18:** Confusion matrix for decision tree classifier.

**Figure 19:** Graphical representation of Table 6.

**Table 1:** Specified parameters of ANN in the proposed work.

Algorithm	Parameter	Value
ANN	Input layer neurons	29
	Hidden layer neurons	15
	Output layer neurons	1
	Activation function on hidden layer	Sigmoid
	Activation function on output layer	Sigmoid
	Number of epochs	1000

**Table 2:** Performance matrices for ANN.

	Precision	Recall	*F*_1_-score
0	0.91	0.94	0.92
1	0.80	0.73	0.76
Overall	0.85	0.83	0.83

**Table 3:** Performance evaluations of random forest classifier.

	Precision	Recall	*F*_1_-score
0	1.00	0.92	0.96
1	0.82	1.00	0.9
Overall	0.91	0.96	0.93

**Table 4:** Performance evaluation of Naïve Bayes classifier.

	Precision	Recall	*F*_1_-score
0	0.65	0.91	0.75
1	0.82	0.45	0.58
Overall	0.81	0.89	0.82

**Table 5:** Performance Metrics for KNN classifier.

	Precision	Recall	*F*_1_-score
0	1.00	0.77	0.87
1	0.61	1.00	0.76
Overall	0.81	0.89	0.82

**Table 6:** Performance metrics for decision tree classifier.

	Precision	Recall	*F*_1_-score
0	1.00	1.00	1.00
1	1.00	1.00	1.00
Overall	1	1	1

**Table 7:** Classification accuracy of proposed method along with other well-known classification methods.

S. No.	Methodology	Classification accuracy
1	SF and ANN [31]	92%
2	DWT and ANN [32]	90%
3	SF, DWT, and ANN [4]	95%
4	SF and KNN [13]	96%
5	Proposed methodology	100%

SF: statistical features; DWT: discrete wavelet transforms; ANN: artificial neural network; KNN: *k*-nearest neighbors' algorithm.

## Data Availability

The dataset is archived from the Harvard University medical website http://www.med.harvard.edu/AANLIB/home.html.
